# The Usage of Designing the Urban Sculpture Scene Based on Edge Computing

**DOI:** 10.1155/2022/9346771

**Published:** 2022-09-14

**Authors:** Junru Zhu

**Affiliations:** Academy of Arts, Sichuan University of Science & Engineering, Zigong, China

## Abstract

To not only achieve the goal of urban cultural construction but also save the cost of urban sculpture space design, EC (edge computing) is combined with urban sculpture space design and planning first. Then it briefly discusses the service category, system architecture, advantages, and characteristics of urban sculpture, as well as the key points and difficulties of its construction, and the layered architecture of EC for urban sculpture spaces is proposed. Secondly, the cloud edge combination technology is adopted, and the urban sculpture is used as a specific function of the edge system node to conduct an in-depth analysis to build an urban sculpture safety supervision system architecture platform. Finally, the actual energy required for implementation is predicted and evaluated, the specific monitoring system coverage is set up, and some equations are made for calculating the energy consumption of the monitored machines according to the number of devices and route planning required by the urban sculpture safety supervision system. An optimization algorithm for energy consumption is proposed based on reinforcement learning and compared with the three control groups. The results show that when the seven monitoring devices cover detection points less than 800, the required energy consumption increases linearly. When the detection devices cover more than 800 detection points, the required energy consumption is stable and varies from 10000 to 12000; that is, when the number of monitoring devices is 7, the optimal number of monitoring points is about 800. When the number of detection points is fixed, increasing the number of monitoring devices in a small range can reduce the total energy consumption. The optimization algorithm based on the reinforcement learning proposal can obtain an approximate optimal solution. The research results show that the combination of edge computing and urban sculpture can expand the function of urban sculpture and make it serve people better.

## 1. Introduction

Urban sculptures are usually independent sculptures in public places such as city streets, squares, railway stations, docks, airports, stadiums, public green spaces, parks, and residential areas. With the development of modern cities, urban environments, and public environments, art has become the focus of urban planning. Educational culture, public environmental art, and urban environmental quality are some of the most important factors. The production of urban sculpture is determined by public artists and decision-makers based on specific environmental factors. In a sense, it is an urban carrier based on the local architectural style and its unique functions. It cannot be replaced by other cultural and artistic forms, especially in cultural and artistic forms that reflect the city's historical and cultural heritage, urban characteristics, and characteristic cultural art form, etc. Urban public art is the local art culture and public space art [1]. In recent years, with the rapid development of higher education in sculpture in China, more and more colleges have offered sculpture-related majors. However, judging from the current urban construction process in China, the sculpture majors offered by existing colleges still cannot meet the needs of urban development, and the quality of sculpture education needs to be improved [2]. It is precise because other professional technology in various aspects has also been applied to this field, such as biotechnology, material science, and technology [3–5].

There are two kinds of definitions approved by the existing research on EC (edge computing). One is to reduce the cost of service delivery and network operation and to provide edge intelligent services in the storage and application of the network edge near data sources. The other is to execute calculations on the edge of the network. The operations of EC need the downlink data from cloud services and the uplink data from the server Internet. And the edge of EC refers to any calculations and network resources between the conversion calculation center paths from data sources to cloud calculations, and it is a continuous system. The emergence of fog computing and EC enlarges the application of cloud computing to pervasive, that is, computationally intensive research [6]. The combination of EC and deep learning based on AI (artificial intelligence) can reduce network risks and protect network safety. Radanliev et al. (2020) studied the relationship between AI and IoT (Internet of Things) and proposed a new dynamic network risk analysis prototype with the edge support of AI [7].

Nowadays, EC and computer technology tend to be applied to urban sculpture and make the style of urban sculpture more diverse and its theme richer. The development of digital technology provides many new technologies and methods for the creation of urban sculpture. Due to the rapid development of communication technology, it is easier for people to acquire cultural specific artistic knowledge, which promotes the internationalization of urban sculpture, making the language and function of urban sculpture more abundant, and changing the manifestation from static to dynamic. This study combines urban sculpture, edge computing (EC), and video structure technology to propose the security monitoring system of urban sculpture scenes and focus on the new forms of urban sculpture in function and service.

Based on the abovementioned analysis, this study combines urban sculpture with edge technology and proposes a safety monitoring system for urban sculpture scenes based on EC and video structure technology. The main contents are as follows: (1). the basic concepts and operation models of EC and the video-structured monitoring system are analyzed, and the concept of edge processor is used to improve the excessive and complex monitoring elements and provide links to the existing security monitoring system of urban sculpture scenes; (2). because of the dispersion and functionality of urban sculpture, a monitoring method combining UAV (unmanned aerial vehicles) with urban sculpture is proposed to improve the performance of the safety monitoring system of urban sculpture; and (3). the model of the safety monitoring system of urban sculpture is constructed, and the experimental data are analyzed to provide a theoretical reference for optimizing the safety monitoring system of urban sculpture. The innovation lies in: (1) the data transmission distance is shortened using EC, and the speed and accuracy of the information in transmission are improved; (2) the energy consumption is calculated and the optimal path is obtained by modeling the path from urban sculpture to UAV under EC; and (3) simulation experiments are carried out in tourist attractions to test the practical function of the system and verify its feasibility.

## 2. Analysis of the Theory and Method of EC Applied to Urban Sculpture

### 2.1. The Relationship between EC and Cloud Computing

EC cannot be applied individually, and it needs the support of various information technologies and technical systems. With the support of IoT, AI, and other technologies, the function and application scope of EC have greatly developed. It is often used to obtain real-time traffic data in cities and metropolitan areas and their surroundings. EC added to the edge application system, the edge storage system, and a series of framework algorithms for application programs and management to meet the needs of different service subjects. These programs and framework algorithms are often combined with blockchain technology to provide safety services for the network [8]. In a sense, it can be regarded as a safety technology that leads to the development of the EC network system. EC can also be combined with cutting-edge technologies. For example, foreign scholars integrate EC and 5G networks to do research, and some scholars apply EC to the UAV, and they have made outstanding achievements in the research [9, 10].

By comparison, EC and cloud computing are mutually complementary [11]. Literally, although cloud computing is powerful, its speed and efficiency of data processing will be subject to constraints and restrictions on different levels. In other words, the energy of cloud computing is limited. Only a certain amount of information can be processed within a certain time limit. However, EC is generated to screen information. Simple information with specific rules is processed at the edge of the network instead of being uploaded to the cloud. In this way, the workload of the cloud can be greatly reduced and work efficiency can be improved. This is the meaning of EC [12].

Common EC and cloud computing application systems are “center + edge” and “no center.” They are adapted to different occasions. Based on its flexibility, the former is mostly used in large systems such as enterprise device management, while the latter is mostly used for simple occasions such as data collection and processing. The combination of the two can bring greater advantages into play, improve efficiency, and guarantee service quality [13].

### 2.2. Application Analysis of EC in Urban Sculpture

EC is powerful and adaptable. It has a wide range of applications in different fields. The application in the urban sculpture industry can also be based on the actual situation, and the core nodes can be flexibly set according to the needs (for example, the data center is the core node, the network device is the core node, the central sculpture is the core node, the platform is the central node, and the system is the core node) [14]. The urban sculpture is considered to have three different application modes at various nodes in cities and industries. They are the urban sculpture as the component node of EC of the urban building system, the urban sculpture as the component node of EC of the urban cultural characteristic dissemination system, and the urban sculpture as the component node of EC of the public service.

When the urban sculpture is used as a component node of EC of the urban sculpture system, the existing urban sculpture resources, and service resources need to be integrated to build the edge urban sculpture system platform [15], and the urban sculptures in a certain area are unified and synchronized management.

City sculptures as the city edge characteristic culture dissemination system calculation, the compositions of the node are the same EC applied to the construction of city characteristic culture when the system, mainly the city cultural buildings, monuments, museums, art museum, the children's palace, data center, financial institutions, knowledge, or data service enterprises such as all kinds of resources integration, formed through the calculation of edge knowledge dissemination system, for the city's cultural construction support [16].

There are four difficulties in the application of urban sculpture. The distribution is a strategic level, capital level, implementation level, and talent reserve level.

At the strategic level, as an emerging technology, EC has powerful functions. But because it is so new, most people are extremely lacking in their understanding of edge technology. The degree of acceptance is even more difficult to talk about. The urban sculpture is a traditional cultural building that has always served the masses. The first problem is how to formulate a reasonable strategic plan to organically integrate urban sculpture and edge technology, to improve the ability of urban sculpture to serve the public with the application of edge technology and ensure that its aesthetics and artistry are not affected, and can be widely accepted by the public [17].

At the financial level, the urban sculpture is located in a superior geographical location, but most of its value comes from the cultural and spiritual values that people attach to it. Such values are established and difficult to change. To make new plans and designs for urban sculptures, whether it is a breakthrough in technical barriers or the use of human resources, new capital injection is required. Therefore, new value points need to be found to bring enough value support to the work [18].

At the implementation level, the fringe transformation of urban sculpture requires a combination of software and hardware. The distribution of urban sculptures is usually numerous and scattered. Moreover, the surrounding environment of the urban sculpture is complicated and the flow of people is large. It takes a lot of time to investigate the situation on the spot during the transformation and planning to ensure that the plan can be implemented.

At the level of talent reserve, after the completion of the fringe city sculpture system, it is necessary to carry out regular inspection and maintenance to ensure its normal work as an edge node. Therefore, a large number of people familiar with sculpture and computer technology are required to enter the reform field and provide service and work, so a large pool of talents in related fields is needed.

### 2.3. System Construction of EC in the Application of Urban Sculpture

To construct the EC construction system of the urban sculpture industry, the composition and links of the edge construction system need to be clarified. That is, city sculptures can provide what services for people, how these services are converted into data, how these data are classified and stratified, how to classify and layer these data, which data and problems should be uploaded to the cloud computing center, what kind of data should be sink to edge computing for direct processing, and which businesses should be the first to start a certain scale of investment and construction [19]. Based on the analysis of these issues, a frame diagram for the construction of the urban sculpture fringe system is proposed, as shown in Figure 1, which mainly includes the core layer, the core application layer, the EC layer, and the front contact layer.

The core layer is the core of the urban sculpture edge system architecture, which mainly includes the basic data center, the infrastructure center, and the basic component center. The core layer is responsible for the management and evaluation of various data collected in the urban sculpture fringe system [20]. For example, in the entire urban sculpture fringe system, the core layer can collect data such as which sculpture location has the highest traffic volume in a certain period, which location has the highest safety incident rate and find out the corresponding reasons to optimize the system. The core application layer consists of five parts, architecture platform, storage deployment, exception management, resource allocation, and data processing. The five applications correspond to different service directions and play a role in data classification and screening [21, 22]. The EC layer is divided into three modules, namely, service applications, cache management, and edge device management. And it is responsible for the preliminary processing and storage of information collected by edge nodes and providing simple feedback to client programs for preliminary management. This is the key to the entire EC architecture. The last one is the front contact layer, which mainly includes data collection and data pre-processing, which is usually combined with the client to directly provide services to customers.

Based on the completion of the construction of the urban sculpture EC framework, it needs to be combined with reality for further application and deepening, and one of the specific modules safety monitoring is selected. The safety monitoring module combines video surveillance and cloud computing technology and uses EC to build a video-structured analysis system platform for the safety monitoring status of urban sculptures. The frame is shown in Figure 2.

The environment where the urban sculpture is located is complex and the flow of people is large. It is difficult and challenging in terms of safety, management, and monitoring. The figure shows that the fringe city sculpture divides the management elements into five key points, namely, characters, methods, devices, environment, and sculpture materials [23]. Characters include clothing, physical state, and movement state. The device includes factors such as the appearance of the vehicle in the entire environment and the state of motion. The material is the characteristics of the sculpture itself, the size and texture, etc., [24]. The specific scene and location are determined through the identification of the sculpture. The method is the processing method of the EC architecture to deal with the outside world obtained through rule modeling. Environment refers to the cognition and analysis of the environment outside the main body of the sculpture. The purpose of safety monitoring is achieved by grasping and analyzing these five key points [25].

The architecture of the entire system needs to use video structured analysis technology as support, which can be divided into two parts, namely, feature modeling and target recognition [26]. Feature modeling refers to the core platform of the urban sculpture edge system, which uses data collected from specific scenes for feature analysis and matching modeling. To cope with the complex environment near the urban sculpture, the modeling is divided into two levels: the basic level and the advanced level. Feature modeling at the basic level mainly refers to the texture of the sculpture and the geometric characteristics of the external environment. The high-level reference refers to the establishment of a database for dynamic information such as human behavior and movement trajectory. Target recognition is to share these databases, summarize the inherent characteristics of the target, match the information that has existed in the scene, make reminders and reflect, and achieve the purpose of avoiding danger and reducing threats.

In terms of data identification and analysis, it is necessary to make the edge nodes have the function of screening, which can determine which data need to be uploaded to the cloud platform and which data can be directly processed by decentralization. Therefore, the data are given two attributes, namely, the delay sensitivity and the strong semantics. The specific analysis of the system is shown in Figure 3.

Figure 3 shows that the key factors of identification analysis are divided into five indicators for the construction of the database in the edge structure of the urban sculpture. The delay-sensitive task is divided into short periodic events, simple events, and urgent events, and it needs to be treated urgently. It usually refers to the safety accident and important note.

In certain scenarios, the edge nodes of the city sculpture are allowed to automatically contact nearby medical institutions for emergency treatment on the spot. Such events usually require timeliness and are suitable for decentralization to EC nodes; strong semantic tasks refer to tasks that are periodic and complex environments that require long-term analysis to make improvements. For example, tourists evaluate the satisfaction of urban sculptures and make suggestions for improvement [27]. Or due to long-term reasons, the traffic section near a certain city sculpture is blocked, and traffic safety incidents occur frequently. This type of data processing is defined as strong semantic data events and needs to be uploaded to the cloud platform to make decisions and analyses.

Strong semantic data will be uploaded, and time-sensitive data will be decentralized. Based on this, the structured analysis platform of urban sculpture cloud edge collaborative video is constructed as shown in Figure 4.

The platform includes four different working modules: data access, intelligent AI platform, container mirroring service, and intelligent edge platform. The data access platform is responsible for classifying and processing the data sent from the edge side. The intelligent AI platform performs big data analysis on the data processed by the data access platform, performs calculations and modeling, and builds a historical database [28]. The container mirroring platform is responsible for backing up various data and performing functional analysis. The intelligent edge platform is responsible for the management, control, and adjustment of all edge nodes to ensure the healthy operation of edge nodes [29].

The last link is the actual contact with tourists. The behavior status of tourists needs a series of monitoring to ensure that there are sufficient data sources and event basis, and it can also provide better services to tourists. The specific architecture is shown in Figure 5.

Various types of vision sensors, such as infrared and thermal sensors, need to be fully utilized and combined with the behavior of tourists near the city sculptures to model their operating conditions across modal characteristics, such as shape, size, and thermal imaging distribution, to perform correlation analysis and adaptive weighted fusion of cross-modal features. A knowledge base of tourist behavior information data based on historical information is constructed to analyze the temporal and spatial topological relationship through feature mapping [30]. Finally, metric learning is used to query and compare the tourist information data knowledge base to realize the joint analysis and comprehensive evaluation of tourist behavior.

### 2.4. Optimal Path Planning Model and Simulation Evaluation under Edge Technology

According to the framework, a deployed mobile EC scene is set up, in which a series of wireless access points, mobile edge micro clouds, and wireless charging points are arranged, and a mathematical model is established to evaluate the structure [31].

Due to the complexity of optimal three-dimensional detection path planning, a heterogeneous detection path planning algorithm is proposed based on reinforcement learning. The equation is as follows:

(1) $$\begin{array}{c} F\left(\text{x},\text{y}\right)=\text{F}\left(\text{x},\text{y}\right)+\text{a}\left(\text{m}+n{\text{max}}_{y1}\text{F}\left(\text{x}1,\text{y}1\right)-\text{F}\left(\text{x},\text{y}\right)\right). \end{array}$$

In (1), x, y is the current state and action of the detection device, x1, y1 is the state of the detection device in the next second, m is a reward for completing an action when the monitoring device is in condition y, x is the reward when the action is completed, a is the learning rate of reinforcement learning, *n* is the recession rate of m. The calculation process of the algorithm is shown in Figure 6.

The energy consumption is calculated by three mathematical modeling algorithms, namely, optimal, greedy, and depth-first search (DFS). They are the members of the control groups, and each of them has its advantages. The relationships between the total energy consumption and the number of device nodes, as well as the number of detection devices, can be obtained by different algorithms. First, the principle of the optimal algorithm is to use IBM ILOG CPLEX to solve the heterogeneous path planning problem realized by AMPL language, and find the optimal solution of the equation by branch and pruning methods. The algorithm helps to obtain the optimal solution accurately and easily, but it also has the disadvantage of long solving time, which is difficult to operate in practical applications and can only be used as a theoretical standard. Second, the greedy algorithm is always the best choice to get the optimal solution at present. That is to say, the algorithm obtains the local optimal solution in a sense, and cannot obtain the overall optimal solution for all problems. The key to getting the optimal solution lies in selecting the appropriate greedy strategy.

The greedy algorithm is a simpler and faster technique for the optimal solution of some problems. It is often solved problems step by step according to the current situation, and makes the best choice from the optimization measures and the best solutions, without considering all possible global situations. This algorithm overcomes the limitation of the time required to make all possible hypotheses, improves efficiency, and reduces the workload. It uses the iterative top-down method to carry out continuous greedy selection. When the selection is made, the original problem is changed into a subproblem. The best solution in the local sense can be achieved by selection. Although the optimal local solution can be obtained after selection, it cannot be ensured that the final optimal solution is global. Each detection device accesses the nearest uncovered area each time until all areas are detected. The greedy algorithm is a simpler and faster technique for some optimal problems. It is characterized by selection step by step, which is often based on the current situation, and makes the optimal choice according to an optimization measure, without considering the overall situation, thus saving a lot of time spent to find the optimal solution from all possible situations. It adopts the top-down method to make successive greedy choices iteratively. Each greedy choice simplifies the problem into a subproblem. Through each choice, an optimal solution to the problem can be obtained. Although it is necessary to ensure that the local optimal solution can be obtained in each step, the overall solution is not necessarily optimal. Here, the greedy algorithm is used to make each detection device access the uncovered area closest to it every time until all areas are detected.

The DFS algorithm is another control algorithm used. The basic idea of DFS is: (1) the vertex *v* is accessed; (2) the depth-first traversal of the graph is performed from the uncovered adjacent point *v* until the vertex in the graph with path *v* is accessed; (3) if a vertex in the graph is not accessed at this time, the depth-first traversal of the graph is performed from an unaccessed vertex until all vertices in the graph are accessed. When it is applied, all regions are connected into a path in the order of depth-first traversal, and then the path is evenly divided into multiple lines. Each detection device is responsible for the detection of one path. In the 1000^*∗*^*∗*1000 map, 100∼1000 detection points, 50 mobile access points, 50 charging devices, and 5∼10 detection devices are randomly set to generate the starting position of the detection device. In addition, different initial power, moving speed, and power consumption rate under different states are set on each device. The parameters are adjusted through two experiments to detect the impact of the number change of the covered areas and detection devices on the energy consumption of the system. Here, a scenic spot is selected to conduct the study. According to the behavior of tourists and the safety accidents in the scenic spot, the statistical results are obtained to verify the feasibility of this study.

## 3. Analysis of Monitoring Energy Consumption Assessment Results

### 3.1. Detect the Relationship between the Number of Nodes and Energy Consumption

Figure 6 shows the change in the total energy consumption of the system when the number of detection nodes that need to be monitored increases from 100 to 1,000. In this set of experiments, the number of detection devices is set to 7.

Figure 7 shows that when the coverage target increases, the proposed reinforcement learning algorithm is compared with the other three algorithms for energy consumption. When the number of monitoring nodes in the coverage area reaches 800, the total mobile energy consumption varies from 10,000 to 12,000. This is because when the targets to be detected are denser, the total movement path changes less, and the required energy consumption is correspondingly reduced. In addition, as a benchmark for comparison, optimal can always get the best solution. Secondly, the planning path of the DFS algorithm is better than the greedy algorithm. This shows that the solution of reinforcement learning is closest to the optimal.

### 3.2. The Relationship between the Number of Detection Devices and Energy Consumption

In addition to the number of detection nodes, another factor that has a greater impact on energy consumption is the number of detection devices. The relationship between the number of detection devices and the required energy consumption is shown in Figure 8 below.

Figure 8 shows the influence of the number of detection devices on the total energy consumption of the system, and the x-coordinate represents the number of detection devices. In this set of experiments, the number of detection points in the total detection coverage area is fixed at 500, and the number of detection devices is between areas (5, 10). Figure 7 shows that when the number of detection devices increases, the total system energy consumption tends to decrease. This is because each detection device only needs to move within a part of the detection area, which reduces the moving distance between the areas.

It is found that reinforcement learning can obtain an approximate optimal solution compared with the other two algorithms. The total energy consumption of the path obtained by the algorithm is the least. In short, the optimal path planning algorithm for monitoring the energy consumption of detection devices based on reinforcement learning proposed can obtain an approximate optimal solution and consumes less energy than the other two algorithms.

### 3.3. Results of System Monitoring

The intelligent monitoring system of urban sculpture based on EC can provide different service functions to tourists according to their historical behavior.  Figure 9 shows the tourists' travel trends from July to December.

Figure 9 shows that the tourists' travel trends in different types of scenic spots are drawn according to the flow at different times in different regions. The data in July show that the weather is hot and tourists tend to travel more watery places, so the flow of tourists around the water is large. As time passes by, their tourism destinations tend to be suburbs and villages, and tourists can plan their trips through instant information provided by edge sculpture nodes. The staff of tourist attractions can also allocate resources reasonably according to the statistical data, which is conducive to improving their work efficiency.

The safety monitoring system of urban sculpture based on EC can monitor and calculate the types of safety accidents in recent months, and the statistical results are shown in Figure 10.

Figure 10 shows that it is an important task to monitor the safety in densely populated areas like the area with urban sculpture. Figure 7 shows the time and type of safety accidents in the tourist attraction where an urban sculpture is located last year. It is found that April and August are the high occurrences of accidents in scenic spot, and the main safety accident is drowning. In addition, November is a month in which fire disasters usually happen. The information is combined with the intelligent monitor system of urban sculpture based on EC can figure out safety and emergency measures in scenic spots.

## 4. Conclusion

The relevant functions and deployment methods of urban sculpture design and planning are constructed from the theoretical and technical levels and combined with the characteristics of the modern urban sculpture industry under the background of EC. Urban sculpture and EC are used to construct an edge system for modern urban sculpture. The general technical route of EC applied to the urban sculpture system is listed, the platform architecture combining urban sculpture and EC is given, and the video joint control analysis technology principle based on the algorithm path planning of optimal, greedy, and DFS and the results of energy consumption analysis is also given. The results of energy consumption analysis have strong practicality. It also provides ideas and references for the application of similar urban architecture and EC. The results show that the intelligent safety monitoring system proposed based on EC can expand the functions of urban sculpture, provide more convenient services for the people, and make the functions of urban sculpture more intelligent and diversified. The relationship between the energy consumption of monitoring devices and the number of the edge node is studied by a simulation experiment. Through the comparison of three algorithms, it is found that as the number of the monitoring nodes covered increases, the energy consumption of the monitoring nodes will gradually increase. The optimal number of detection nodes should be maintained at about 800. The proposed reinforcement algorithm can obtain the approximate optimal solution. The simulation results show that the intelligent monitoring system of urban sculpture based on EC can improve the practical value of urban sculpture and provide better services for people.

Since multiple fields are involved, the combination of urban sculpture and EC is still in the process of exploration, and the research stays at the theoretical framework and technical level of system construction. Although the simulation experiment was carried out, further research is still needed due to the constraints of research funding and experience. In the follow-up research, more environmental factors will be considered to make the research better and applicable in real life.

## Figures and Tables

**Figure 1:** Urban sculpture edge system architecture.

**Figure 2:** Analysis of the safety monitoring system.

**Figure 3:** Cloud edge collaborative architecture.

**Figure 4:** Urban sculpture edge supervision platform (A-E in the figure represent target detection, target re-recognition, behavior recognition, semantic segmentation, scene recognition).

**Figure 5:** Video joint control and analysis technology principle.

**Figure 6:** Calculation process of reinforcement learning.

**Figure 7:** Relationship between the number of detection nodes and energy consumption.

**Figure 8:** Relationship of energy consumption and the number of detection devices.

**Figure 9:** Tourists' travel trends in different types of scenic spots.

**Figure 10:** Statistics of safety accidents.

## Data Availability

The raw data supporting the conclusions of this article will be made available by the authors, without undue reservation.

## References

[1] Tsagkaropoulos A., Verginadis Y., Compastié M., Apostolou D., Mentzas G. (2021). Extending TOSCA for edge and fog deployment support. *Electronics*.

[2] Florita N. J. B., Senatin A. N. M., Zabala A. M. A., Tan W. M. (2020). Opportunistic LoRa-based gateways for delay-tolerant sensor data collection in urban settings. *Computer Communications*.

[3] Zhang J., Lu C., Cheng G. (2021). A blockchain-based trusted edge platform in edge computing environment. *Sensors*.

[4] Le T. (2021). Multi-hop routing under short contact in delay tolerant networks. *Computer Communications*.

[5] Amos P., Li P., Wu W., Wang B. (2021). Computation efficiency maximization for secure UAV-enabled mobile edge computing networks. *Physical Communication*.

[6] Zhou E., Zhang J., Dai K. (2020). Research on task and resource matching mechanism in the edge computing network. *International Core Journal of Engineering*.

[7] Radanliev P., De Roure D., Walton R. (2020). Artificial intelligence and machine learning in dynamic cyber risk analytics at the edge. *SN Applied Sciences*.

[8] Silva N., Pullar R. C., Pintado M. E., Vieira E., Moreira P. R. (2018). Biotechnology for preventive conservation: development of bionanomaterials for antimicrobial coating of outdoor sculptures. *Studies in Conservation*.

[9] Ksentini A., Frangoudis P. A. (2020). Toward slicing-enabled multi-access edge computing in 5G. *IEEE Network*.

[10] Mukherjee A., Dey N., De D. (2020). Edge Drone: QoS aware MQTT middleware for mobile edge computing in opportunistic Internet of Drone Things. *Computer Communications*.

[11] Li W., Wang S., Koo C. (2021). A real-time optimal control strategy for multi-zone VAV air-conditioning systems adopting a multi-agent based distributed optimization method. *Applied Energy*.

[12] Zhang X., Cao Z., Dong W. (2020). Overview of edge computing in the agricultural internet of things: key technologies, applications, challenges. *IEEE Access*.

[13] Chen Z., Xiao N., Han D. (2020). Multilevel task offloading and resource optimization of edge computing networks considering UAV relay and green energy. *Applied Sciences*.

[14] Tritschler N., Dugenske A., Kurfess T. (2021). An automated edge computing-based condition health monitoring system: with an application on rolling element bearings. *Journal of Manufacturing Science and Engineering*.

[15] Li J., Zhou G., Tian T., Li X. (2021). A new cooling strategy for edge computing servers using compact looped heat pipe. *Applied Thermal Engineering*.

[16] Wang W., Huang H., Xue L., Li Q., Malekian R., Zhang Y. (2021). Blockchain-assisted handover authentication for intelligent telehealth in multi-server edge computing environment. *Journal of Systems Architecture*.

[17] Peng K., Nie J., Kumar N. (2021). Joint optimization of service chain caching and task offloading in mobile edge computing. *Applied Soft Computing*.

[18] Mohan L., Farooq D., Rajesh S. (2021). GEESE: edge computing enabled by UAV. *Pervasive and Mobile Computing*.

[19] Liu X., Jiang Y. Z. (2021). A real-time detection method for abnormal data of internet of things sensors based on mobile edge computing. *Mathematical Problems in Engineering*.

[20] Fu Y., Yang X., Yang P. (2021). Energy-efficient offloading and resource allocation for mobile edge computing enabled mission-critical internet-of-things systems. *EURASIP Journal on Wireless Communications and Networking*.

[21] Nithya K. (2020). Geographic routing in WSN for measuring coverage constraints and energy consumption in cloud environments. *International Journal of Innovative Technology and Exploring Engineering*.

[22] Balamuralidhar N., Tilon S., Nex F. (2021). MultEYE: monitoring system for real-time vehicle detection, tracking and speed estimation from UAV imagery on edge-computing platforms. *Remote Sensing*.

[23] Qin N., Li B., Li D., Jing X., Du C., Wan C. (2021). Resource allocation method based on mobile edge computing in smart grid. *IOP Conference Series: Earth and Environmental Science*.

[24] Zhang H., Liu Z., Zhang Y. (2021). Research on deployment method of edge computing gateway based on microservice architecture. *IOP Conference Series: Earth and Environmental Science*.

[25] Liu C., Su X., Li C. (2021). Edge computing for data anomaly detection of multi-sensors in underground mining. *Electronics*.

[26] Pahič R., Lončarević Z., Gams A., Ude A. (2021). Robot skill learning in latent space of a deep autoencoder neural network. *Robotics and Autonomous Systems*.

[27] Zhang G., Peng G. H. (2019). Research on the stabilization effect of continuous self-delayed traffic flux in macro traffic modeling. *Physica A: Statistical Mechanics and Its Applications*.

[28] Cui M., Zhang H., Huang Y., Xu Z., Zhao Q. (2021). A fountain-coding based cooperative jamming strategy for secure service migration in edge computing. *Wireless Networks*.

[29] Guo S., Zhang K., Gong B., He W., Qiu X. (2021). A delay-sensitive resource allocation algorithm for container cluster in edge computing environment. *Computer Communications*.

[30] Li n (2020). Construction of landscape architecture art design based on streaming media data processing. *International Journal of Arts and Technology*.

[31] Chowdary K. M., Kuppili V. (2021). Enhanced clustering and intelligent mobile sink path construction for an efficient data gathering in wireless sensor networks. *Arabian Journal for Science and Engineering*.

